The article "Pre-treatment DWI as a predictor of overall survival in locally advanced pancreatic cancer treated with Cyberknife radiotherapy and sequential S-1 therapy" was retracted in 2018. Reason: duplicate publication.

# Pre-treatment DWI as a predictor of overall survival in locally advanced pancreatic cancer treated with Cyberknife radiotherapy and sequential S-1 therapy

**DOI:** 10.1186/s40644-018-0139-7

**Published:** 2018-02-22

**Authors:** Yu Zhang, Xiaofei Zhu, Denghui Liu, Jiaqi Song, Huojun Zhang, Jianping Lu

**Affiliations:** 1 Department of Radiology, Changhai Hospital Affiliated to the Second Military Medical University, Changhai Road 168, Yangpu district, Shanghai, 200433 People’s Republic of China; 2 Department of Oncology Radiation, Changhai Hospital Affiliated to the Second Military Medical University, Changhai Road 168, Yangpu district, Shanghai, 200433 People’s Republic of China; 3 Department of Orthopedics, No. 113 Hospital of People’s Liberation Army, East Zhongshan Road 377, Jiangdong District, Ningbo, 315000 People’s Republic of China; 4 Department of health statistics, Second Military Medical University, Xiangyin Road 800, Yangpu district, Shanghai, 200433 People’s Republic of China

**Keywords:** Cyberknife, Prognosis, Locally advanced pancreatic cancer, Radiotherapy, Diffusion weighted imaging

## Abstract

**Background:**

To identify the value of the pre-treatment apparent diffusion coefficient (ADC) derived from diffusion weighted imaging (DWI) in predicting the overall survival (OS) for locally advanced pancreatic cancer (LAPC) treated with Cyberknife followed by sequential S-1 chemotherapy.

**Methods:**

Patients with UICC-T4 LAPC who underwent DWI scan (3.0 Tesla) using two b-values (0, 600 s/mm^2^) in our center between 2015 and 2017 were enrolled. Mean ADCs of the region of interest (ROI) drawn manually on DWI imaging were measured by two independent radiologists at an interval of 1 month. The association between prognostic factors and patient survival was determined using univariate and multivariate analyses. Cox proportional hazard model was used for identification of independent prognostic factors of OS.

**Results:**

A total of 41 patients (28 males and 13 females) were included, with a median age of 64 years, with 5 patients (3 males and 2 females) lost. The median OS was 11.7 months (range 2.8–23.3) among all 41 patients. The 1-year OS was 46% (95% CI 30%–62%). Univariate and multivariate analyses indicated that pre-treatment ADC value (HR 10.652, *P* = 0.0093), age (HR 0.952, *P* = 0.015), CA19–9 (HR 1.001, *P* = 0.0022) and administration of S-1 (HR 0.128, *P* = 0.0002) were independent predicting factors of OS.

**Conclusion:**

The mean ADC value of the primary tumor on pre-treatment DWI imaging was an independent predictor of OS in patients with LAPC receiving Cyberknife followed by sequential S-1.

## Background

Patients with locally advanced pancreatic cancer (LAPC) are generally no longer candidates for curative surgeries and chemoradiotherapy is the standard therapeutic option [1]. Stereotactic body radiation therapy, with its advantages of lower incidences of radiation-induced toxicity, higher accuracy and better efficacy compared with conventional radiotherapy, has gained momentum in the management of advanced-stage pancreatic malignancies [2]. S-1, as an important chemotherapeutic agent in pancreatic cancer, which has been proved with equal survival benefits comparing to the standard gemcitabine with no higher incidences of the adverse effects [2]. Currently, few encouraging results investigating the safety and efficacy of combination therapy of S-1 and the other medications have been published. Thus, the combination of S-1 and radiotherapy has also gained popularity in the treatment of pancreatic cancer.

The article "Pre-treatment DWI as a predictor of overall survival in locally advanced pancreatic cancer treated with Cyberknife radiotherapy and sequential S-1 therapy" was retracted in 2018. Reason: duplicate publication.

Random diffusion of water molecules (i.e. the Brownian motions) could be illustrated by diffusion weighted imaging (DWI), an approach of functional imaging, to generate contrast in magnet resonance images. DWI is important in depicting tumor tissues in vivo and non-invasively. The mobility of water could be determined in a quantitative way by apparent diffusion coefficient (ADC). Besides, the modifications of water diffusion induced by any factors could also by detected by ADC. In addition to existing clinical and pathologic prognostic factors, ADC can serve as a useful imaging biomarker through better characterization of individual tumor biology. Therefore, this study aims to investigate the value of pre-treatment DWI-MRI in predicting OS in patients with LAPC undergoing Cyberknife followed by sequential S-1.

## Methods

### Patients

This prospective study was approved by the Changhai Hospital Ethics Committee (CHEC-2016-032-01). Written informed consent was obtained from all participants prior to MRI imaging examinations. Histopathological diagnosis with fine-needle aspiration guided by endoscopic ultrasound was preferred for all patients suspected of pancreatic cancer. The planned period of follow-up for each patient was 2 years. All included patients should meet the following criteria: 1) Patients with pancreatic cancer and no distant metastasis prior to MRI scan; 2) patients without MRI contraindications, including claustrophobia, implanted metal foreign body and certain type of cardiac pacemaker; 3) patients with no known allergy to gadolinium-based contrast agent; 4) patients without any anticancer treatment prior to Cyberknife. Therefore, consecutive 41 UICC-T4 patients (28 males and 13 females) with a median age of 64 years (range: 44–80 years) received Cyberknife followed by two to three courses of sequential S-1 in our center during 2015 to 2017.

The article "Pre-treatment DWI as a predictor of overall survival in locally advanced pancreatic cancer treated with Cyberknife radiotherapy and sequential S-1 therapy" was retracted in 2018. Reason: duplicate publication.

### MRI

Prior to radiotherapy, MRI scan was performed on a 3.0-Tesla MR scanner (Signa HDxt V16.0, GE Healthcare, Milwaukee, USA) with an eight-element phased array coil and transverse respiratory triggered technique. Table 1 showed the main MRI parameters and the order of scanning sequences. At the end of the study, T1-weighted imaging gradientrecalledecho (T1WI GRE) was performed with a gadopentetate dimeglumine injection (contrast media, 0.2 ml/kg, a rate of 3 mL/s; physiological saline, the same amount and injection rate).

**Table 1:** Scanning parameters of MR sequences

Sequences	TR/TE (msec)	FOV (cm **×** cm)	Matrix	Thickness/gap (mm)	Flip angle(^0^)	No of Slices	NEX^a^	Bandwidth (KHz)	Speed factor
MRCP	7000/1200	30 **×** 30	288 **×** 288	50/0	–	6	0.92	31.25	–
T1WI GRE	4.3/1.3	44 **×** 40	320 × 224	5 mm volume	12	–	1	166.67	1.79
T2WI	6316/72	38 **×** 38	330 **×** 192	5/1	90	22	2	83.33	1.25
DWI	6000/56.5	38 **×** 30	96 **×** 128	5/1	90	25	1/4^a^	250	2
Contrast-enhanced T1WI GRE	4.3/1.3	44 **×** 40	320 × 224	5 mm volume	12	–	1	166.67	1.79

^a^NEX = 1 for DWI at b_0_, NEX = 4 for DWI at b_600_

*MRCP* Magnetic resonance cholangiopancreatography, *T2WI T2* Weighted imaging

*T1WI GRE T1* Weighted imaging gradientrecalledecho, *DWI* Diffusing weighted imaging

### Stereotactic body radiation therapy procedures and chemotherapy regimens

Stereotactic body radiation therapy was delivered by Cyberknife (Accuracy, Sunnyvale, CA, USA). Patients were immobilized in the supine position with a vacuum bag. Spiral computed tomography (CT) was performed with a slice thickness of 1.5 mm. Gross tumor volume (GTV) was delineated as a radiographically evident gross disease by contrast CT. At the discretion of the physician, clinical target volume (CTV) encompassing areas of the potential subclinical disease spread was also designated. In most cases, the CTV equaled to GTV. A 2-5 mm expansion margin was included to determine the planning target volume (PTV). The prescription dose varied from 30–36Gy in five to six fractions. Normal tissue constraints were observed according to the American Association of Physicists in Medicine guidelines in TG-101 [3], as presented in Tables 2 and 3. The prescription dose was devised to be the isodose line encompassing > 97% of the planning target volume (PTV). No more than 3% of the PTV received < 93% of the prescription dose. The X sight Spine Tracking System and fiducials were used in a 4 Dimension-CT treatment simulation.

**Table 2:** Parallel organs and threshold doses

Parallel organs	Threshold doses (five fractions)	Minimum critical volume below threshold
Liver	21 Gy	700 cm^3^
Kidney	17.5 Gy	200 cm^3^

The article "Pre-treatment DWI as a predictor of overall survival in locally advanced pancreatic cancer treated with Cyberknife radiotherapy and sequential S-1 therapy" was retracted in 2018. Reason: duplicate publication.

**Table 3:** Serial organs and threshold doses

Serial organs	Threshold doses (five fractions)	Max point dose	Max critical volume above threshold
Spinal cord	23 Gy	30 Gy	0.35 cm^3^
Duodenum	18 Gy	32 Gy	5 cm^3^
Bowel	19.5 Gy	35 Gy	5 cm^3^
Stomach	18 Gy	32 Gy	10 cm^3^
Esophagus	19.5 Gy	35 Gy	5 cm^3^
Colon	25 Gy	38 Gy	20 cm^3^

S-1 is the prodrug of 5-fluorouracil (5-FU), which comprises of tegafur, gimeracil (dihydropyrimidine dehydrogenase inhibitor) and oteracil (inhibitor of phosphorylation in the gastrointestinal tract), with a ratio of 1:0.4:1. It has been demonstrated to be effective in the management of pancreatic cancer [4]. After radiotherapy, 2 or 3 cycles of S-1 were sequentially given. One cycle consisted of 28 days of oral S-1 at a dose of 80 mg/m^2^ for twice a day. Cycles were separated by a 14-day interval.

### Radiologic parameters

DWI-data was post-processed on a workstation (Function V9.4.05, GE AW 4.4, GE Healthcare). The ADC was calculated at the single slice with the longest tumor diameter using the following algorithm: ADC = 1/b In (S_0_/S), where b referred to the b-factor (600 s/mm^2^), S_0_ represented the signal intensity for b = 0 s/mm^2^ image and S as the signal intensity at b = 600 s/mm^2^ image. ADC represented the measured mean ADC, using two b -values (0, 600 s/mm^2^).

### Radiologic analysis

Region of interest (ROI) indicated the largest possible single-slice area at the level of the maximum diameter of the tumor [5].Based on T2-weighted imaging(T2WI) with exclusion of pancreatic ducts, cystic lesions and necrotic areas, the ROI parameter was simultaneously calculated on the ADC map using a workstation by a standard software package (Function V9.4.05, GE AW 4.4, GE Healthcare). The borders of the tumor on DWI image were determined after the radiologists had reviewed pre-treatment T2WI and T1WI images. The areas of ROI ranged from 101mm^2^ to 2970 mm^2^.

### Statistical analysis

OS was evaluated from the initial date of radiotherapy to the death of patients. All variables were expressed as mean ± standard deviation (SD). Intraclass correlation (ICC, value and strength of correlation: 0–0.20: poor correlation; 0.21–0.40: fair correlation; 0.41–0.60: moderate correlation; 0.61–0.80: good correlation; 0.81–1.00: excellent correlation) [6] was estimated to evaluate the consistency of ADCs between two investigators. When the level of consistency was acceptable, the result rated by the first radiologist doctor was adopted. Log-rank test was conducted to evaluate the association of patient survival and tumour location, S-1, presence or absence of biliary stent, and other treatment. Cox regression was employed to identify potential factors predictive of OS.*P* < 0.05 indicated a statistical significant level. All statistical analyses were conducted by SAS 9.4 software (SAS Institute Inc., Cary, NC, USA).

The article "Pre-treatment DWI as a predictor of overall survival in locally advanced pancreatic cancer treated with Cyberknife radiotherapy and sequential S-1 therapy" was retracted in 2018. Reason: duplicate publication.

## Results

### Patients’ characteristics

Among 41 enrolled patients, 34 had pancreatic head carcinoma with 7 lesions located in the body and tail of the pancreas. The median tumor diameter was 3.7 cm (range: 1.6–8.2 cm). 16 patients had biliary stent implanted, and S-1 was given to 32 patients. 11 patients received other treatment after metastasis, of who 2 had transcatheter arterial chemoembolization (TACE), 3 took herbal antineoplastic agents (traditional Chinese medicine), 2 underwent ablation therapy, 3 received gemcitabine and ^125^I seed was implanted in 1 patient. These 11 patients were not further categorized according to the treatment they had due to a small sample. Five patients were totally lost of follow-up without any medical records after treatment.

### Interobserver variability of ADC values

The typical axial MRI images and ADC map for ADC measurement were demonstrated in Fig. 1. ICC showed good consistency between both investigators. For the ADC values, the mean difference and the 95% confidence interval of the mean difference (limits of agreement) between two readers were 0.00293 [95%CI: -0.01202, 0.01787] (ICC, 0.987).

**Fig. 1:** A 41-year-old female patient with histological proven pancreatic adenocarcinoma in the head of the pancreas. The images showed the lesion with clearly demarcated hyperintensity area compared with the surrounding normal tissues on DWI images. Axial contrast-enhanced MRI image depicted a hypointense lesion in the head of the pancreas (**a**); Axial T2WI (**b**); freehand ROIs were drawn along the high signal intensity border of the tumor with obtained DWI images (b = 600 s/mm^2^, (**c**) to cover the largest possible single-slice area. ADC (DWI) map (**d**)

### Independent predictors of OS

The median OS was 11.7 months and the 1-year OS rate was 46% (95% CI: 30%–62%). Log-rank test analysis showed that there was no significant correlation between OS and tumour location, presence or absence of biliary stent as well as other treatment. However, the initiation of S-1 correlated with OS. Orally taken S-1 provided better prognosis (*P* = 0.018, Fig. 2). Furthermore, though OS did not correlate with tumor location and other treatment, patients with other treatment had a tendency towards prolonged OS compared with those who did not (*P* = 0.230, Fig. 3). Patients with tumor in the body and tail of the pancreas tended to have a better OS, compared with those with lesions in the head of the pancreas (*P* = 0.261 Fig. 4). Multivariate analysis showed that pre-treatment ADC value (HR 10.652, *P* = 0.0093), age (HR 0.952, *P* = 0.015), pre-treatment CA19–9 (HR 1.001, *P* = 0.0022) and S-1 regimen (HR 0.128, *P* = 0.0002) were predictive of OS. In other words, a lower pre-treatment ADC value, an older age, a lower level of pre-treatment CA19–9 and initiation of S-1 were all associated with a better survival (Table 4**,** Figs. 5 and 6).

The article "Pre-treatment DWI as a predictor of overall survival in locally advanced pancreatic cancer treated with Cyberknife radiotherapy and sequential S-1 therapy" was retracted in 2018. Reason: duplicate publication.

**Fig. 2:** The survival curves showed significant difference between S-1 and no S-1 taken (*P* = 0.018)

**Fig. 3:** The survival curves showed patients with other treatment had a tendency towards prolonged OS, compared to those who did not (*P* = 0.230)

**Fig. 4:** Patients with tumor in the body and tail of the pancreas tended to have a better OS, compared to those with tumor in the head of the pancreas (*P* = 0.261)

**Table 4:** Cox regression result for ADC (DWI)

Variables	*β*	*χ* ^2^	*P*	HR	%95 CI	
					Low	Up
Age	−0.0493	5.9134	0.0150	0.952	0.915	0.990
S-1	−2.0594	13.9914	0.0002	0.128	0.043	0.375
ADC	2.3657	6.7595	0.0093	10.652	1.790	63.378
CA 19–9	0.0012	9.3611	0.0022	1.001	1.000	1.002

**Fig. 5:** MRI images of histological proven pancreatic cancer in 73-year-old male patient without oral S-1 chemotherapy. The ADC value of the lesion was 2.06 × 10^− 3^ mm^2^/s and the pre-treatment CA19–9 level was 1200 U/ml. The OS was 185 days. Axial precontrast T1WI (**a**); Axial T2WI (**b**); Axial contrast-enhanced T1WI (**c**); DWI image (b = 600 s/mm^2^, (**d**));freehand ROIs were drawn along the high signal intensity border of the tumor with obtained DWI images (600 s/mm^2^, (**e**)) to cover the largest possible single-slice area. Zoomed-in ADC (DWI) map with a high ADC (**f**)

**Fig. 6:** MRI images of histological proven pancreatic cancer in 56-year-old female patient with a lower ADC (1.08 × 10^− 3^ mm^2^/s), orally taken S-1 and a lower pre-treatment CA19–9 level (339.9 U/ml). The OS was 522 days. Axial precontrast T1WI (**a**); Axial T2WI (**b**); Axial contrast-enhanced T1WI (**c**); DWI image (b = 600 s/mm^2^, (**d**)); freehand ROIs were drawn along the high signal intensity border of the tumor with obtained DWI images (b = 600 s/mm^2^, (**e**)) to cover the largest possible single-slice area. Zoomed-in ADC (DWI) map with a lower ADC (**f**)

## Discussion

DWI is an important approach of functional imaging and has been widely used in clinical radiology. ADC, by measuring the Brownian motion of water molecules in tumor tissues, is a promising quantitative biomarker in the field of oncologic radiology [7–9]. To our knowledge, DWI has been used to predict and monitor the outcomes of many types of tumors, such as rectal, brain and cervical cancer [10–13].These pre-treatment predictions allow clinicians to optimize treatment strategies for individual patients and avoid unnecessary costs, side effects and treatment delays. However, few studies have investigated the use of pre-treatment DWI in predicting the survival of patients with LAPC receiving Cyberknife and sequential S-1 therapy.

The article "Pre-treatment DWI as a predictor of overall survival in locally advanced pancreatic cancer treated with Cyberknife radiotherapy and sequential S-1 therapy" was retracted in 2018. Reason: duplicate publication.

As is known to all, characterized by excessive cell proliferation and resistance to cell death, malignant cancers can often present with increased cellularity. The increased cell density may break the normal balance between the intra- and extracellular compartments within tissues, reducing extracellular volumes, and eventually resulting in alterations in the water movement, which would be well reflected in diffusion measurements [14]. Pancreatic cancer usually consists of a large number of tumor parenchymal cells and fibrous tissues derived from the pancreatic stellate cells. Consequently, the ADC value of pancreatic cancer is lower than that of normal pancreatic tissues. Previous studies have reported a negative correlation between tumor cellularity and ADC values in pancreatic malignancies [15, 16], which was probably due to restricted diffusion of water molecules resulting from increased cellularity. However, the negative association between ADC values and cellularity of PDAC warrants further study, primarily because the normal pancreas tissues are found to be composed of abundant serous acinar cells [17–19], and the fact that the ADC of normal pancreatic tissues is higher than that of PDAC should be considered. Thus, cellularity difference cannot be solely attributable to the ADC differences between PDAC and the surrounding normal pancreatic tissues and between different lesions [15]. Additionally, difference in water diffusivity between tissues should also be ascribed to other mechanisms. The correlation between ADC and tumor fibrosis is controversial. Klauss et al. reported increased values of the parameter D, the true diffusion component of tissue, in denser fibrous tissues [20]. Others reported no correlations between ADC values and the degree of tumor fibrosis [21, 22]. Muraoka et al. found that the mean ADC value was significantly higher in tumors with loose fibrotic tissues than that with dense fibrotic tissues, and ADC value correlated well with the proportion of collagenous fibers [23]. Ma et al. found that the ADC value of PDAC negatively correlated with the proportion of fibrotic contents and fibroblast activation protein staining scores [24]. In addition, poor vascularity of PDAC was attributed to the activation of abundant fibrotic stroma in the tumor microenvironment, resulting attenuation of microvessel density compared to the normal pancreatic tissues [25]. In other words, the ADC level of pancreatic malignancies is affected by various factors: cellularity, the extent of fibrosis and vascularity and etc.

The article "Pre-treatment DWI as a predictor of overall survival in locally advanced pancreatic cancer treated with Cyberknife radiotherapy and sequential S-1 therapy" was retracted in 2018. Reason: duplicate publication.

In the present study, we found that a lower pre-treatment ADC value was significantly associated with better OS, which was consistent with previous similar studies on liver and kidney malignancies [11, 26–28]. However, this should be interpreted with cautions because various factors would affect the value of ADC: Firstly, highly proliferating tumor cells resulted in increased cellularity, which implied a lower level of ADC. Those proliferating tumor cells are sensitive to radiotherapy and chemotherapy [29, 30].Secondly, loss of cell membrane integrity of the malignant tissue indicating a more aggressive phenotype prior to treatment could result in higher pre-treatment ADC and a worse OS [26].Thirdly, lesions with higher ADC levels may contain more dense fibrotic tissues, leading to a poor prognosis [20]. Additionally, abundantly dense fibrotic tissues in tumor contributed to poor vascularity [27], resulting in less delivery of chemotherapeutic agents to these areas. Finally, lesions with higher ADC can contain necrotic pooling which may predispose the tumor cells to a more hypoxic and acidic environment, which may diminish the effectiveness of chemotherapy.

S-1 has emerged as an important chemotherapeutic drug in pancreatic cancer recently. Many studies have demonstrated that S-1, with its favorable oral administration, was not inferior to gemcitabine in terms of OS, PFS, and rates of adverse effects [31]. Therefore, S-1 can serve as an alternative to gemcitabine for locally advanced or metastatic pancreatic cancer. In addition, neoadjuvant chemoradiotherapy with S-1 could probably be in favor of down-staging and decreased incidences of surgical complications [32, 33]. It also indicated that neoadjuvant chemoradiotherapy with S-1 was beneficial to potential candidates for further radical surgeries due to the increased OS [33]. In our study, we found that S-1 were significantly associated with prolonged OS in patients with LAPC, which showed the good clinical efficacy of S-1. Patients with lower levels of pre-treatment CA19–9 had longer OS, which was consistent with previous studies [34, 35] . In addition, better prognosis was found in older patients than that in younger ones. We also found that tumor in the body and tail of the pancreas and those with other treatment had a better OS, which could be attributed to the fact that prescription doses for the tumor in the head of the pancreas might be compromised due to adjacent organs compared with those for the tumor in the body and tail of the pancreas and that pancreatic head tumours are more likely to have the involvement of important adjacent organs and effect of interventional procedures and chemotherapy. It was also showed that there was no significant association found between OS and gender, tumor diameter, as well as presence or absence of biliary stents.

The article "Pre-treatment DWI as a predictor of overall survival in locally advanced pancreatic cancer treated with Cyberknife radiotherapy and sequential S-1 therapy" was retracted in 2018. Reason: duplicate publication.

The optimal recommended respiratory triggered approach [36] was used in our abdominal MR imaging to avoid the influence of breathing motion artifacts in ADC measurement, affected by identifying ROI, b-values, field strength, data post-processing models, and respiratory compensation acquisition and etc. Furthermore, DWI MR imaging provides information on perfusion and diffusion simultaneously in any organs. It has been clarified that the choice of b value played an important role in which of these contributions [37, 38], at the same time, to achieve a balance between motion artifacts and the signal-to-noise ratio (SNR), the optimal b-value (600 s/mm^2^) for abdominal lesions was used [39].

Nevertheless, there were some limitations in the current study. Firstly, the eligible patient number is relatively small regarding the statistical significance identified between the OS of the patients and predictors such as tumor location and other treatment. Future studies with larger sample size is warranted for the validation of our preliminary results. Secondly, we investigated the tumor mean ADC out of many quantitative imaging parameters such as min ADC and SUV, since they had been used as representative parameters to predict clinical outcomes for various cancers.

## Conclusion

In summary, the pre-treatment ADC value was a significant predictor of OS in patients with LAPC treated with Cyberknife followed by sequential S-1.

## References

[1] Su TS, Liang P, Lu HZ, Liang JN, Liu JM, Zhou Y (2015). Stereotactic body radiotherapy using CyberKnife for locally advanced unresectable and metastatic pancreatic cancer. World J Gastroenterol.

[2] Zhu X, Ju X, Cao F, Fang F, Qing S, Shen Y (2016). Safety and efficacy of stereotactic body radiation therapy combined with S-1 simultaneously followed by sequential S-1 as an initial treatment for locally advanced pancreatic cancer (SILAPANC) trial: study design and rationale of a phase II clinical trial. BMJ Open.

[3] Benedict SH, Yenice KM, Followill D, Galvin JM, Hinson W, Kavanagh B (2010). Stereotactic body radiation therapy: the report of AAPM task group 101. Med Phys.

[4] Ueno H, Okusaka T, Ikeda M, Takezako Y, Morizane C (2005). An early phase II study of S-1 in patients with metastatic pancreatic cancer. Oncology.

The article "Pre-treatment DWI as a predictor of overall survival in locally advanced pancreatic cancer treated with Cyberknife radiotherapy and sequential S-1 therapy" was retracted in 2018. Reason: duplicate publication.

[5] Ma C, Liu L, Li J, Wang L, Chen LG, Zhang Y (2016). Apparent diffusion coefficient (ADC) measurements in pancreatic adenocarcinoma: a preliminary study of the effect of region of interest on ADC values and interobserver variability. J Magn Reson Imaging.

[6] Cohen J (1968). Weighted kappa: nominal scale agreement with provision for scaled disagreement or partial credit. Psychol Bull.

[7] Sun YS, Zhang XP, Tang L, Ji JF, Gu J, Cai Y (2010). Locally advanced rectal carcinoma treated with preoperative chemotherapy and radiation therapy: preliminary analysis of diffusion-weighted MR imaging for early detection of tumor histopathologic downstaging. Radiology.

[8] Hein PA, Kremser C, Judmaier W, Griebel J, Pfeiffer KP, Kreczy A (2003). Diffusion-weighted magnetic resonance imaging for monitoring diffusion changes in rectal carcinoma during combined, preoperative chemoradiation: preliminary results of a prospective study. Eur J Radiol.

[9] Kim SH, Lee JM, Hong SH, Kim GH, Lee JY, Han JK (2009). Locally advanced rectal cancer: added value of diffusion-weighted MR imaging in the evaluation of tumor response to neoadjuvant chemo- and radiation therapy. Radiology.

[10] Chenevert TL, McKeever PE, Ross BD (1997). Monitoring early response of experimental brain tumors to therapy using diffusion magnetic resonance imaging. Clin Cancer Res.

[11] Dzik-Jurasz A, Domenig C, George M, Wolber J, Padhani A, Brown G (2002). Diffusion MRI for prediction of response of rectal cancer to chemoradiation. Lancet.

[12] McVeigh PZ, Syed AM, Milosevic M, Fyles A, Haider MA (2008). Diffusion-weighted MRI in cervical cancer. Eur Radiol.

[13] Ho JC, Allen PK, Bhosale PR, Rauch GM, Fuller CD, Mohamed AS (2017). Diffusion-weighted magnetic resonance imaging as a predictor of outcome in cervical cancer after Chemoradiation. Int J Radiat Oncol Biol Phys.

[14] Paran Y, Bendel P, Margalit R, Degani H (2004). Water diffusion in the different microenvironments of breast cancer. NMR Biomed.

[15] Heid I, Steiger K, Trajkovic-Arsic M, Settles M, Esswein MR, Erkan M (2017). Co-clinical assessment of tumor cellularity in pancreatic cancer. Clin Cancer Res.

[16] Wang Y, Chen ZE, Yaghmai V, Nikolaidis P, McCarthy RJ, Merrick L (2011). Diffusion-weighted MR imaging in pancreatic endocrine tumors correlated with histopathologic characteristics. J Magn Reson Imaging.

[17] Conrad R, Castelino-Prabhu S, Cobb C, Raza A (2013). Cytopathology of the pancreatobiliary tract-the agony, and sometimes, the ease of it. J Gastrointest Oncol.

[18] Biankin AV, Waddell N, Kassahn KS, Gingras MC, Muthuswamy LB, Johns AL (2012). Pancreatic cancer genomes reveal aberrations in axon guidance pathway genes. Nature.

The article "Pre-treatment DWI as a predictor of overall survival in locally advanced pancreatic cancer treated with Cyberknife radiotherapy and sequential S-1 therapy" was retracted in 2018. Reason: duplicate publication.

[19] Moffitt RA, Marayati R, Flate EL, Volmar KE, Loeza SG, Hoadley KA (2015). Virtual microdissection identifies distinct tumor- and stroma-specific subtypes of pancreatic ductal adenocarcinoma. Nat Genet.

[20] Klauss M, Gaida MM, Lemke A, Grunberg K, Simon D, Wente MN (2013). Fibrosis and pancreatic lesions: counterintuitive behavior of the diffusion imaging-derived structural diffusion coefficient d. Invest Radiol.

[21] Rosenkrantz AB, Matza BW, Sabach A, Hajdu CH, Hindman N (2013). Pancreatic cancer: lack of association between apparent diffusion coefficient values and adverse pathological features. Clin Radiol.

[22] Noda Y, Goshima S, Tanaka K, Osada S, Tomita H, Hara A (2016). Findings in pancreatic MRI associated with pancreatic fibrosis and HbA1c values. J Magn Reson Imaging.

[23] Muraoka N, Uematsu H, Kimura H, Imamura Y, Fujiwara Y, Murakami M (2008). Apparent diffusion coefficient in pancreatic cancer: characterization and histopathological correlations. J Magn Reson Imaging.

[24] Ma W, Li N, Zhao W, Ren J, Wei M, Yang Y (2016). Apparent diffusion coefficient and dynamic contrast-enhanced magnetic resonance imaging in pancreatic cancer: characteristics and correlation with histopathologic parameters. J Comput Assist Tomogr.

[25] Erkan M, Hausmann S, Michalski CW, Fingerle AA, Dobritz M, Kleeff J (2012). The role of stroma in pancreatic cancer: diagnostic and therapeutic implications. Nat Rev Gastroenterol Hepatol.

[26] Koh DM, Scurr E, Collins D, Kanber B, Norman A, Leach MO (2007). Predicting response of colorectal hepatic metastasis: value of pretreatment apparent diffusion coefficients. AJR Am J Roentgenol.

[27] Cui Y, Zhang XP, Sun YS, Tang L, Shen L (2008). Apparent diffusion coefficient: potential imaging biomarker for prediction and early detection of response to chemotherapy in hepatic metastases. Radiology.

[28] DeVries AF, Kremser C, Hein PA, Griebel J, Krezcy A, Ofner D (2003). Tumor microcirculation and diffusion predict therapy outcome for primary rectal carcinoma. Int J Radiat Oncol Biol Phys.

[29] Hatakenaka M, Nakamura K, Yabuuchi H, Shioyama Y, Matsuo Y, Ohnishi K (2011). Pretreatment apparent diffusion coefficient of the primary lesion correlates with local failure in head-and-neck cancer treated with chemoradiotherapy or radiotherapy. Int J Radiat Oncol Biol Phys.

[30] Lu Y, Jansen JF, Stambuk HE, Gupta G, Lee N, Gonen M (2013). Comparing primary tumors and metastatic nodes in head and neck cancer using intravoxel incoherent motion imaging: a preliminary experience. J Comput Assist Tomogr.

[31] Ueno H, Ioka T, Ikeda M, Ohkawa S, Yanagimoto H, Boku N (2013). Randomized phase III study of gemcitabine plus S-1, S-1 alone, or gemcitabine alone in patients with locally advanced and metastatic pancreatic cancer in Japan and Taiwan: GEST study. J Clin Oncol.

The article "Pre-treatment DWI as a predictor of overall survival in locally advanced pancreatic cancer treated with Cyberknife radiotherapy and sequential S-1 therapy" was retracted in 2018. Reason: duplicate publication.

[32] Breslin TM, Hess KR, Harbison DB, Jean ME, Cleary KR, Dackiw AP (2001). Neoadjuvant chemoradiotherapy for adenocarcinoma of the pancreas: treatment variables and survival duration. Ann Surg Oncol.

[33] Laurence JM, Tran PD, Morarji K, Eslick GD, Lam VW, Sandroussi C (2011). A systematic review and meta-analysis of survival and surgical outcomes following neoadjuvant chemoradiotherapy for pancreatic cancer. J Gastrointest Surg.

[34] Gu YL, Lan C, Pei H, Yang SN, Liu YF, Xiao LL (2015). Applicative value of serum CA19-9, CEA, CA125 and CA242 in diagnosis and prognosis for patients with pancreatic cancer treated by concurrent Chemoradiotherapy. Asian Pac J Cancer Prev.

[35] Sugiura T, Uesaka K, Kanemoto H, Mizuno T, Sasaki K, Furukawa H (2012). Serum CA19-9 is a significant predictor among preoperative parameters for early recurrence after resection of pancreatic adenocarcinoma. J Gastrointest Surg.

[36] Kartalis N, Loizou L, Edsborg N, Segersvard R, Albiin N (2012). Optimising diffusion-weighted MR imaging for demonstrating pancreatic cancer: a comparison of respiratory-triggered, free-breathing and breath-hold techniques. Eur Radiol.

[37] Thoeny HC, De Keyzer F, Boesch C, Hermans R (2004). Diffusion-weighted imaging of the parotid gland: influence of the choice of b-values on the apparent diffusion coefficient value. J Magn Reson Imaging.

[38] Le Bihan D, Breton E, Lallemand D, Aubin ML, Vignaud J, Laval-Jeantet M (1988). Separation of diffusion and perfusion in intravoxel incoherent motion MR imaging. Radiology.

[39] Koc Z, Erbay G (2014). Optimal b value in diffusion-weighted imaging for differentiation of abdominal lesions. J Magn Reson Imaging.

